# Artificial Intelligence Pulse Coupled Neural Network Algorithm in the Diagnosis and Treatment of Severe Sepsis Complicated with Acute Kidney Injury under Ultrasound Image

**DOI:** 10.1155/2021/6761364

**Published:** 2021-07-20

**Authors:** Fu Ying, Shuhua Chen, Guojun Pan, Zemin He

**Affiliations:** ^1^Department of Emergency Medicine, Changzhou Cancer Hospital, Changzhou 213000, Jiangsu, China; ^2^Department of Intensive Care Unit, Changzhou Cancer Hospital, Changzhou 213000, Jiangsu, China

## Abstract

The objective of this study was to explore the diagnosis of severe sepsis complicated with acute kidney injury (AKI) by ultrasonic image information based on the artificial intelligence pulse coupled neural network (PCNN) algorithm. In this study, an algorithm of ultrasonic image information enhancement based on the artificial intelligence PCNN was constructed and compared with the histogram equalization algorithm and linear transformation algorithm. After that, it was applied to the ultrasonic image diagnosis of 20 cases of severe sepsis combined with AKI in hospital. The condition of each patient was diagnosed by ultrasound image performance, change of renal resistance index (RRI), ultrasound score, and receiver operator characteristic curve (ROC) analysis. It was found that the histogram distribution of this algorithm was relatively uniform, and the information of each gray level was obviously retained and enhanced, which had the best effect in this algorithm; there was a marked individual difference in the values of RRI. Overall, the values of RRI showed a slight upward trend after admission to the intensive care unit (ICU). The RRI was taken as the dependent variable, time as the fixed-effect model, and patients as the random effect; the parameter value of time was between 0.012 and 0.015, *p*=0.000 < 0.05. Besides, there was no huge difference in the ultrasonic score among different time measurements (*t* = 1.348 and *p*=0.128 > 0.05). The area under the ROC curve of the RRI for the diagnosis of AKI at the 2^nd^ day, 4^th^ day, and 6^th^ day was 0.758, 0.841, and 0.856, respectively, which was all greater than 0.5 (*p* < 0.05). In conclusion, the proposed algorithm in this study could significantly enhance the amount of information in ultrasound images. In addition, the change of RRI values measured by ultrasound images based on the artificial intelligence PCNN was associated with AKI.

## 1. Introduction

Acute kidney injury (AKI) refers to a clinical syndrome caused by a rapid decline in renal function within a short period that led to various etiologies. It can occur in people without previous kidney disease or in patients with existing chronic kidney disease [1]. AKI is a common emergency and critical illness, and its prevalence in ordinary hospitalized patients is 3–5%. Moreover, the prevalence of AKI is as high as 30–50% in the intensive care unit (ICU) [2]. Although blood purification technology is constantly being updated, the mortality rate of patients with AKI has not been markedly reduced, which is an acute and critical disease in kidney disease [3]. The early course of AKI is reversible, but its treatment window is narrow. Once the injury period is entered, the incidence of death or uremia will exceed 30% [4]. Therefore, the early diagnosis of AKI, the improvement of the treatment effect of AKI, and the reduction of the mortality rate of AKI have a very critical scientific value and clinical significance.

In patients with AKI, Doppler ultrasound (DU) is often adopted to determine the renal resistance index (RRI) of the renal interlobular artery [5]. Bragato et al. [6] reported that RRI could assess the renal function of patients with AKI. Most importantly, RRI is correlated with renal vascular resistance, renal vascular compliance, renal blood flow, oxygen partial pressure, renal interstitial pressure, and other aspects, most of which are risk factors for AKI, so it can be used to effectively evaluate AKI [7]. In recent years, Kim et al. [8] have shown that DU can be used for the early diagnosis of kidney injury in patients with severe sepsis. DU can evaluate the ultrasound score of patients in a semiquantitative manner, and the operation is simple. However, there are few reports on the application of DU to evaluate the renal function of patients with severe sepsis and AKI [9].

The artificial intelligence pulse coupled neural network (PCNN) algorithm can construct neuron mapping into a phase-based model, which carries information not only the pulse frequency but also a sign of the transmission channel [10]. The artificial intelligence PCNN makes the way of selecting communication routes and the construction of computers simpler and more effective. Compared with other neural network models, the PCNN is more practical. The artificial intelligence PCNN uses a single-layer neural network model, which can be directly applied to image segmentation, pattern recognition, and image fusion without training [11]. Lotfinejad et al. [12] have adopted the artificial intelligence PCNN to image processing, finding that the PCNN had the advantages of constant signal strength, constant rotation, and constant scale under weak connection conditions.

In this study, the artificial intelligence PCNN algorithm was compared with the histogram equalization algorithm and linear transformation algorithm. Then, they were applied to the ultrasound images of 20 patients with severe sepsis combined with AKI, aiming to explore the ultrasound image characteristics of severe sepsis combined with AKI. Therefore, it could provide a reliable reference basis for early diagnosis and early treatment of clinical AKI patients.

## 2. Materials and Methods

### 2.1. Research Objects

In this study, 20 patients diagnosed with severe sepsis and AKI in the hospital from December 2018 to October 2019 were selected as the research objects. Besides, all of them underwent ultrasound examinations. There were 13 males and 7 females, with an average age of 48.69 ± 12.47 years. This study had been approved by the ethics committee of the hospital, and the research objects included in this study and their family members signed the informed consent forms.

The criteria for inclusion were defined to include patients who met the diagnostic criteria for severe sepsis, with tissue hypoperfusion and renal dysfunction caused by sepsis, can undergo the assisted breathing treatment through a ventilator, and were 18–75 years old.

The criteria for exclusion were defined to include patients who were younger than 18 years old, were in the recovery period of AKI, were accompanied with obstructive renal failure, intraabdominal hypertension, arrhythmia, and other diseases that would affect the value of RRI, suffered from chronic renal insufficiency, and were combined with heart, spleen, and cardiovascular and cerebrovascular diseases.

### 2.2. Construction of Ultrasound Images Based on Artificial Intelligence Pulse Coupled Neural Network Algorithm

Figure 1 shows the artificial intelligence PCNN algorithm model. When the PCNN processed the images, it was a single-layer two-dimensional network. The number of neurons was consistent with the number of pixels in the output image. The pixel intensity of the gray-scale image was the excitation condition of the neuron. The surrounding input neurons connected with each output neuron to form an image processing system based on the PCNN algorithm. In this study, a threshold *F*_*i*,*j*_ was constructed to represent the Mach band effect. The Laplacian operator $L=\left[\begin{array}{ccc} -1 & -1 & -1\\ -1 & 6 & -1\\ -1 & -1 & -1 \end{array}\right]$ was convolved with the gray-scale image of the input excitation, so that the size of the threshold *F*_*i*,*j*_ was redefined as follows.

(1) $$\begin{array}{c} F_{i,j}\left(0\right)=\text{BPG}-{\text{CPG}}_{i,j}. \end{array}$$

In equation (1), BPG represents the gray value of the brightest pixel of the original image input, and CPG_*i*,*j*_ represents the gray value of the neuron (*i*, *j*) point image after convolution processing. The network output of the PCNN was transformed into the gray-scale excitation value perceived by the network to obtain the final enhanced image. Besides, the equation was as follows.

(2) $$\begin{array}{c} \text{EIG}=\text{In}\left(\text{BPG}\right)-\tau \left(S\left(i,j\right)-1\right). \end{array}$$

In equation (2), EIG represents the gray value of the enhanced image, BPG represents the brightest pixel gray value of the original image input, *S*(*i*, *j*) represents the ignition timing of the neuron (*i*, *j*), and *τ* represents the attenuation constant.

The specific steps of the PCNN algorithm included the following.

Step 1: first, the parameters of the PCNN were set, and the number of cycles was set as *M*, so that all neurons were in the inhibited state. The gray value of the PCNN algorithm image was calculated to construct the matrix *S* of neuron ignition time and determine the threshold *F*_*i*,*j*_. The specific algorithm flow steps were expressed in the following equations.
  (3) $$\begin{array}{c} F_{i,j}\left[m\right]=S_{i,j}\left[m\right], \end{array}$$
  (4) $$\begin{array}{c} R_{i,j}\left[m\right]=W_{L}\sum VY\left[m\right], \end{array}$$
  (5) $$\begin{array}{c} U\left[m\right]=F_{i.j}\left[m\right]\left(1+\alpha R_{i,j}\left[m\right]\right), \end{array}$$
  (6) $$\begin{array}{c} Y_{i,j}\left[m\right]=1,\;\text{if }U\left[m\right]>F_{i,j}\left[m\right]\text{ or otherwise,} \end{array}$$
  (7) $$\begin{array}{c} F_{i,j}\left[m\right]=\exp\left(-\tau \right)\times F\left(i,j\right)+W_{E}\times Y\left(i,j\right). \end{array}$$
In the above equations, the PCNN parameters *α*=0.2, *τ*=0.7, *W*_*L*_=1, *W*_*F*_=278, *F*_*i*,*j*_ represents the dynamic threshold, *m* represents the number of iterations, *S*(*i*, *j*) represents the ignition timing of the neuron (*i*, *j*), *R*_*i*,*j*_[*m*] represents the feedback input of the neuron (*i*, *j*)'s *m*^th^ iteration, *Y*_*i*,*j*_[*m*] represents the feedback output of the neuron (*i*, *j*)'s *m*^th^ iteration, *α* represents the strength constant of links between synapses, *U*[*m*] represents the internal activity item, *W*_*L*_ represents the amplitude constant of *F*_*i*,*j*_[*m*], and *W*_*F*_ represents the threshold decay time coefficient.
Step 2: the neuron ignited at a certain moment and could output a pulse to record the ignition moment in *S*. The threshold of the neuron was taken as the maximum value to inhibit the occurrence of reignition. What is more, the equations are given as follows:
  (8) $$\begin{array}{c} S_{i,j}\left[m\right]=m,\;\text{if }E_{i,j}\left[m\right]\;=1,\;{\text{mark}}_{i,j}\left[m\right]=0, \end{array}$$
  (9) $$\begin{array}{c} {\text{mark}}_{i,j}\left[m\right]=\infty i,\;\text{if }E_{i,j}\left[m\right]=1,\text{ otherwise }0, \end{array}$$
  (10) $$\begin{array}{c} E_{i,j}\left[m\right]=\infty ,\;\text{if }Y_{i,j}\left[m\right]=1. \end{array}$$
Step 3: if one of the neurons ignited, the final output value was 1, and the gray value of the image could be enhanced according to equation (2).
Step 4: all gray values were processed, so it would be ended; otherwise, return to Step 2.

### 2.3. Ultrasound Scoring Standards for Severe Sepsis Patients Combined with Kidney Injury

The diagnostic criteria of severe sepsis combined with AKI in this study referred to the diagnostic criteria of severe sepsis in the 2012 Scientific Steering Committee (SSC) guidelines [13]. The patients received the DU examinations, and their ultrasound images were saved in ultrasound equipment, which was scored (DU scoring) by 3 physicians who were specially trained in emergency and critical ultrasound. Using a 0–3 semiquantitative scoring standard, the ultrasound scoring was as follows. 0 point indicated that no renal blood vessels could be detected, 1 point meant that a few blood vessels could be observed in the renal hilum, 2 points showed that interlobular blood vessels could be observed in the renal parenchyma, and 3 points presented that the renal arcuate artery level could be found in the kidney.

### 2.4. Renal Ultrasound Examination

Within 24 hours of entering ICU, each patient was given with renal ultrasound examination when the hemodynamics was stable. The patients were detected through ultrasound once a day for 7 consecutive days until they left the ICU. Besides, the ultrasound examinations were conducted by the physicians who were specially trained in emergency and critical ultrasound and were not involved in the treatment. The Vivid i portable Doppler ultrasound (produced by GE, USA) was employed to explore the kidneys on both sides of the patient, and a 5 Hz ultrasound probe was adopted to observe whether the kidneys had contusions or hematomas and whether there was damage to the bilateral renal arteries. Finally, RRI was measured, first on the right kidney and then on the left.

The measurement of RRI was as follows. First, the protruding probe was used for the detection of the patient's abdomen, and the long axial section of the kidney was intercepted from the posterolateral position of the two-dimensional ultrasound. Doppler was applied to identify the renal vessels to locate an interlobular artery. Then, the minimum Doppler sampling gate 3–6 mm and minimum pulse repetition frequency (PRF) where graphics did not overlap were set to obtain 4–6 consecutive similar spectra. Moreover, statistical measurements of the peak systolic velocity (SV) and the minimum diastolic velocity (DV) were made to calculate the RRI of each spectrum. In addition, the RRI for each spectrum could be calculated by the following equation.

(11) $$\begin{array}{c} \text{RRI}=\frac{\left(\text{SV}-\text{DV}\right)}{\text{SV}}. \end{array}$$

In equation (11), SV represents the peak flow velocity in the systolic period and DV represents the lowest diastolic flow rate. Furthermore, the average value of the RRI was taken after 4–6 measurements.

### 2.5. Statistical Methods

The test data processing was carried out using SPSS20.0 statistical software. The measurement data were expressed as the mean ± standard deviation ($\bar{x}$ ± *s*), and the *t*-test was used for the comparison of the average values between each group. The count data were represented by the percentage (%), and the *χ*^2^ test was used. The RRI at different time points was used as the diagnostic evaluation test to draw the ROC and determine the optimal critical value of RRI for the diagnosis of AKI. What is more, the AUC of ROC was compared between each time point. In addition, *p* < 0.05 indicated that the difference was statistically substantial.

## 3. Results

### 3.1. Ultrasound Image Quality Evaluation Results Based on Artificial Intelligence Pulse Coupled Neural Network Algorithm

Figure 2 shows the ultrasound images of equalization, linear transformation algorithm, and artificial intelligence PCNN algorithm. The results showed that histogram equalization was a global image enhancement algorithm that could extend the gray scale of low-brightness ultrasound images, and eventually, overenhancement occurred. The transformation function adopted by the linear transformation algorithm was relatively simple, and the final imaging effect was not ideal. The artificial intelligence PCNN algorithm proposed in this study not only considered the global information but also enhanced the local information. After enhancement, the gray value of the ultrasound image was evenly distributed near the gray value sensitive to the human eye, and the overall image effect was suitable for direct observation with naked eyes.

The histograms of AKI, histogram equalization, linear transformation algorithm, and artificial intelligence PCNN algorithm are shown in Figure 3. To verify the effectiveness of the artificial intelligence PCNN algorithm, it was compared with the equalization method and the linear transformation algorithm. It was found that the histogram of the equalization method was mainly concentrated in a large area and the distribution was relatively uniform, but there was the enhancement after the image was enhanced, and the overall image effect was not very good. The linear transformation algorithm was mainly concentrated in the darker area, the enhancement was not obvious, and the overall effect was not good. The histogram of the artificial intelligence PCNN algorithm was relatively evenly distributed, and each gray level was retained, with significantly enhanced ultrasound image information, which was convenient for the medical diagnosis of AKI. Therefore, it showed that the artificial intelligence PCNN algorithm was the best among the three algorithms in enhancing the information content of the ultrasonic images.

### 3.2. General Information of Patients with Severe Sepsis Combined with Acute Kidney Injury

Figure 4 shows the general data of patients with severe sepsis combined with AKI. In this study, there were a total of 20 severe sepsis patients with AKI, including 13 males (65%) and 7 females (35%), with an average age of 48.69 ± 12.47 years. The patient's injury severity score (ISS) was 32.5 ± 8.9 points, and the acute physiology and chronic health status score II (APACHE II score) was 16.2 ± 9.4 points. Among them, 7 cases (35%) were injured by road traffic accidents, followed by 4 cases (20%) injured by falling from a height, 3 cases (15%) injured by heavy objects, 2 cases (10%) injured by beatings, 3 cases (15%) with machine strangulation injuries, and 1 case (5%) with explosion injury. Finally, 3 cases died, 1 case died of hemorrhage at the trauma site, 1 case died of severe sepsis, and 1 case died of multiple organ failure after severe head injury.

### 3.3. Ultrasound Image Performance Characteristics Based on Artificial Intelligence Pulse Coupled Neural Network Algorithm

The ultrasound images based on the artificial intelligence PCNN algorithm are shown in Figure 5. Ultrasound is an important method for diagnosing AKI and judging the prognosis. Whether it was glomerular sclerosis, renal tubular atrophy, interstitial fibrosis, or inflammation, ultrasound imaging showed enhanced cortical echo. The cortex became thinner and the echo was enhanced; the renal cortex and the medulla echo were not demarcated; the focal cortex was thinned; the echo was enhanced, with the uniform structure, and the renal parenchyma and the renal sinus could not be distinguished by naked eyes; the cortical echo was enhanced, and the upper pole of the kidney was unclear; the cortex echoes enhanced, and the kidneys enlarged; the lower pole of the kidney was lacerated, and the subcapsular fluid was accumulated.

### 3.4. Changes in Ultrasound Renal Resistance Index in Severe Sepsis Patients Combined with Acute Kidney Injury

Figure 6 includes the two graphs showing the changing trend of ultrasound RRI in patients with severe sepsis combined with AKI. According to the changing trend in the figure, there were obvious individual differences in RRI; on the whole, RRI indicated a slight upward trend after the patient entered ICU.

The analysis results of the linear mixed model of RRI and time are presented in Table 1. The RRI was used as the dependent variable, time was used as a fixed-effect model, and the patient was treated as a random effect. The parameter value of time was 0.012–0.015, *p* < 0.001, which verified that RRI would increase over time. Among them, 2 patients had AKI after entering ICU, 1 patient had a marked increase in RRI after AKI, and 1 patient showed a significant downward trend.

### 3.5. Ultrasound Scores of Severe Sepsis Patients Combined with Acute Kidney Injury

The ultrasound scores of patients with severe sepsis and AKI are shown in Figure 7. Over time, the ultrasound scores of patients with severe sepsis and AKI were mainly distributed in 2 points.

Table 2 reveals the analysis results of the linear mixed model of RRI and time. The ultrasound score was used as the dependent variable, time was a fixed-effect, patient time was used as a fixed-effect model, and the patient was taken as a random effect. The parameter value of time was 0.001–0.015, *p*=0.128 > 0.05, indicating that there was no substantial difference in the ultrasound scores of patients with severe sepsis complicated with AKI (*t* = 1.348 and *p*=0.128 > 0.05).

### 3.6. ROC Curve Analysis of Renal Resistance Index at Different Time Points in the Diagnosis of Severe Sepsis with Acute Kidney Injury

Figure 8 shows the ROC curves of the RRI for the diagnosis of AKI on the 2^nd^ day, 4^th^ day, and 6^th^ day after entering the ICU. Besides, the AUC values of ROC for RRI diagnosis of AKI at different time points were analyzed, and the analysis results are given in Table 3. The patient with AKI was defined as a positive index as 1, and the ROC of RRI on the 2^nd^ day, 4^th^ day, and 6^th^ day after entering ICU was drawn to the diagnosis of AKI. Furthermore, the values of AUC were 0.758, 0.841, and 0.856 in turn, which were all greater than 0.5 (*p* < 0.05).

## 4. Discussion

AKI is a complication of traumatic diseases, and the common risk factors for its occurrence include the severity of the trauma, the degree of bleeding, shock, traumatic inflammation, and severe sepsis [14]. In this study, 20 patients with severe sepsis combined with AKI were included, and there were no marked differences in gender, age, and ISS.

DU has the advantages of high reproducibility and noninvasiveness, which is extensively applied in the field of acute and critical illness and has shown a good diagnostic value in the assessment of renal trauma [15–17]. DU can quantitatively determine the resistance index of renal interlobular arteries. Xia et al. [18] confirmed that RRI could predict the occurrence of AKI in the state of severe sepsis. According to the changing trend of the RRI within 1–7 days after entering the ICU, there were obvious individual differences in RRI [19]. On the whole, the RRI had a slight upward trend after entering the ICU. The RRI, time, and the patient were taken as the dependent variable, a fixed-effect model, and a random effect, respectively. The parameter value of time was 0.012–0.015, *p* < 0.001, verifying that RRI would rise over time.

The AUC of ROC for the diagnosis of AKI was drawn on the 2^nd^ day, 4^th^ day, and 6^th^ day of entering the ICU [20]. The patient with AKI was defined as a positive index as 1, and the ROC curves of RRI on the 2^nd^ day, 4^th^ day, and 6^th^ day after entering the ICU were drawn to the diagnosis of AKI. What is more, the values of AUC were 0.758, 0.841, and 0.856 in sequence, all greater than 0.5 (*p* < 0.05), suggesting that the AUC of ROC drawn in this study had high accuracy. Thus, RRI could be used as a predictive index of AKI.

## 5. Conclusion

The artificial intelligence PCNN algorithm in this study was compared with histogram equalization algorithm and linear transformation algorithm, which were adopted for the ultrasound images of 20 patients with severe sepsis and AKI. The results disclosed that the artificial intelligence PCNN algorithm proposed in this study not only considered the global information of ultrasound images but also enhanced the local information of ultrasound images. In addition, the changes in RRI measured by ultrasound images were related to AKI. The shortcomings of this study are that the time is limited, the number of samples collected is small, and the patient observation time is only about 1 week. It is impossible to observe the changes of RRI before and after kidney injury and during the recovery period of AKI. Further research is needed in the later period. All in all, the artificial intelligence PCNN algorithm has a significant effect on ultrasound image enhancement, thereby providing a reference theoretical basis for the diagnosis of severe sepsis with AKI.

## Figures and Tables

**Figure 1:** Artificial intelligence PCNN algorithm model.

**Figure 2:** The ultrasound images of (a) histogram equalization, (b) linear transformation algorithm, and (c) artificial intelligence PCNN algorithm.

**Figure 3:** The histograms of (a) severe sepsis with AKI, (b) histogram equalization, (c) linear transformation method, and (d) artificial intelligence PCNN algorithm.

**Figure 4:** General data of patients with severe sepsis combined with AKI. (a) Ratio of male to female in severe sepsis patients with AKI. (b) Types of injury in severe sepsis patients with AKI.

**Figure 5:** Ultrasound images based on artificial intelligence PCNN algorithm. (a) Ultrasound image of renal cortex thinning and echo enhancement. (b) Ultrasound image of renal cortex and medulla echo being unclear. (c) Cortical echo enhancement and an ultrasound image of renal enlargement. (d) Ultrasound image of renal inferior pole laceration and subcapsular effusion.

**Figure 6:** Trend chart of ultrasound RRI changes in severe sepsis patients combined with AKI. (a) The changing trend of RRI of randomly selected cases. (b) The changing trend of average RRI of patients on ultrasound.

**Figure 7:** Ultrasound scores of severe sepsis patients combined with AKI. ^*∗*^Compared to DU = 2 points, *p* < 0.05.

**Figure 8:** The ROC curves of the RRI on the 2^nd^ day, 4^th^ day, and 6^th^ day after entering the ICU for the diagnosis of AKI. The AUC values were 0.758, 0.841, and 0.856, respectively, which were all greater than 0.5 (*p* < 0.05).

**Table 1:** Analysis of the linear mixed model of RRI and time effect.

Parameters	Standard error	95% CI	*t*	*P*
Time	0.002	0.012–0.015	12.348	<0.001
Intercept	0.007	0.638–0.758	64.854	<0.001

**Table 2:** Linear mixed model analysis of ultrasound scores and time effect.

Parameters	Standard error	95% CI	*t*	*P*
Time	0.003	0.001–0.015	1.348	0.128
Intercept	1.225	1.126–2.154	13.238	<0.001

**Table 3:** Analysis of the AUC of the ROC curves of RRI at different time points in the diagnosis of AKI.

Time	AUC	95% CI	Standard error	*P* value
The 2^nd^ day	0.758	0.526–0.974	0.148	1.241
The 4^th^ day	0.841	0.540–0.985	0.134	1.126
The 6^th^ day	0.8526	0.623–1.000	0.012	1.364

*Note*. The *P* value was compared with the value of AUC (0.5).

## Data Availability

No data were used to support this study.
